# Video Analysis and System Construction of Basketball Game by Lightweight Deep Learning under the Internet of Things

**DOI:** 10.1155/2022/6118798

**Published:** 2022-03-15

**Authors:** Tianyu Yang, Congmeng Jiang, Pengfei Li

**Affiliations:** ^1^Department of Physics, Northeastern University at Qinhuangdao, Qinhuangdao 066004, China; ^2^Postgraduate School, Northeastern University at Qinhuangdao, Qinhuangdao 066004, China; ^3^Department of Information Engineering, Qinhuangdao Vocational and Technical College, Qinhuangdao 066100, China

## Abstract

With the explosive growth of sports video data on the internet platform, how to scientifically manage this information has become a major challenge in the current big data era. In this context, a new lightweight player segmentation algorithm is proposed to realize the automatic analysis of basketball game video. Firstly, semantic events are expressed by extracting group and global motion features. A complete basketball game video is divided into three stages, and a basketball event classification method integrating global group motion patterns and domain knowledge is proposed. Secondly, a player segmentation algorithm based on lightweight deep learning is proposed to detect basketball players, segment the players, and finally extract players' spatial features based on deep learning to realize players' pose estimation. As the experimental results indicate, when a proposed 2-stage classification algorithm is used to classify the videos, the accuracy of identifying layup, the shooting, and other 2-pointers are improved by 21.26% and 6.41%, respectively. And the accuracy of average events sees an improvement of 2.74%. The results imply that the 2-stage classification based on event-occ is effective. After comparing the four methods of classifying players, it is found that there is no significant difference among these four methods about the accuracy of segmenting. Nevertheless, when judged with the time that these methods take separately, FCN-CNN (Fully Convolutional Network-Convolutional Neural Network) based on superpixels has overwhelming advantages. The event analysis method of basketball game video proposed here can realize the automatic analysis of basketball video, which is beneficial to promoting the rapid development of basketball and even sports.

## 1. Introduction

In the current environment, the technical revolution is booming. As the vital driving force of this industrial revolution, computer network technology is constantly changing people's way of life and work, pushing human society into an intelligent new one with human-machine fusion and mutual sharing the creating. As the core technology of the current technological revolution, applying deep learning into the sports industry is the need of time [1, 2]. Due to the rapid development of the internet, various big sports events are widely broadcast. Simultaneously, people's attention on these events is seeing a continuous uprising. However, with the wide broadcast of videos related to sports events, how to scientifically manage the data of sports video is becoming a problem that arises researchers' focus [3]. Videos related to sports include many kinds of sports games, such as single-player games, single/double confrontation games, and two-team confrontation games. There is not much background interference and obstacle in the videos related to single/double confrontation games such as table tennis and badminton, nor as to the complexity of players' movements. However, confrontation games involve many people, and players' movements are complicated. And it is difficult to analyze videos related to such kinds of sports events, like football, basketball, and ice-ball [4–6].

In nearly a few years, the sports events video has drawn lots of attention from researchers, especially the complex videos related to basketball. In the past, when analyzing the basketball game video, the broadcaster needs to identify different events of players according to acoustic characteristics and text. However, along with the development of deep learning, some scholars adopted the technology into the analysis of basketball game video [7–10]. Ravi et al. analyzed a single shooting video based on a deep learning algorithm. At first, they used VGG (Visual Geometry Group)-16 to extract the spatial features of movements information and sampling frames. Then they combined spatial features with timing features with Action VLAD Pooling [11]. Zhao et al. captured the tracks of basketball in data from a real basketball game, based on a mixed density network framework and dual-direction recursion network. Besides, new tracks of sampling data can be obtained. Hence, the application can determine the shooting position and shooting time, providing significant help to athletes [12]. Batista et al. proposed a hierarchical model for behavior recognition of multi person activity video. The model decomposed human behavior into multilevel detail information, thus fully expressing the interactive relationship between individuals in the scene [13]. Cooper studied highly structured multiperson activity recognition and proposed an algorithm framework based on the fusion of low-order time-domain individual distribution relationship and probability model. However, the method of handmade features cannot make full use of the interaction between each individual [14]. Due to the complexity of the scale of the basketball game and the problem of mutual occlusion between players, it will be relatively difficult to extract the key players. What is worse, the background in the basketball game is very complex, which will lead to a sharp increase in the amount of calculation and cause target confusion.

The spatial features of global motion patterns are extracted based on Convolutional Neural Network (CNN), and the player area is segmented based on the Fully Convolutional Network- Convolutional Neural Network (FCN-CNN) method of superpixel clustering, to identify the player's posture. The proposed FCN-CNN player segmentation algorithm based on superpixel filters out the complex background around the player, which is more conducive to subsequent attitude estimation. It realizes the automatic analysis of basketball video, thus assisting the coach to formulate tactics, the players to analyze actions, and the video viewers to quickly search interested video segments, and promoting the rapid development of basketball and even sports.

## 2. Basketball Events Analysis Based on the Deep Learning Algorithm

### 2.1. The Algorithm and the Total Framework to Estimate Player's Posture

Figure 1 illustrates the overall classification framework in basketball game videos, based on multidomain knowledge and Global and Collective Motion Patterns (GCMPs) proposed here.

As Figure 1 reveals, the two-stage event classification is mainly divided into five overall types of event classification and two detailed types of event classification. The five overall types of event classification are based on event-occ video segment and combined with Global and Collective Motion Pattern Deep features of images in the sequential video frame (GCMP-DF-SVF) information, such as 2-pointer, 3-pointer, penalty ball, and steal. The fine classification of the two types of events is based on the preevent video segment and combined with GCMP-DF-SVF information. The above two classification stages are realized by Convolutional Neural Network and Long Short-Term Memory (CNN + LSTM) to extract information and express the sequence and spatial characteristics of GCMPs. Then the event results are predicted based on the postevent video segment. Finally, the event prediction results are combined with the classification results to form the final prediction results.

### 2.2. Classification of Semantic Events

Due to the similarity between the two types of event classification and the five types of event classification, the current work mainly introduces the five types of event classification framework.  Figure 2 demonstrates the framework diagram based on GCMPs event classification.

#### 2.2.1. Expression of Spatial Features of GCMPs

In the analysis of basketball game video, the traditional method is to extract video features manually, but the extracted video features are difficult to express the deep semantic features in the image. Here, based on the application of CNN in deep features learning, the spatial features of GCMPs are extracted by CNN.  Figure 3 signifies the specific framework [15].

Figure 3 manifests that the neural network contains five convolution layers and three full connection layers, and the pooling layer is only added to the convolution layers 1, 2, and 5. Sign “fc” represents the full connection layer. The number of neurons in the three full connection layers is 4096, 4096, and 5, respectively. The number of neurons in the full connection layer 8 is adjusted from 1000 to 5 to realize the five classifications of events such as snatching, shooting, and penalty. Equation (1) illustrates the size relationship between the input layer and the output layer.

(1) $$\begin{array}{c} Y_{i}=\frac{\left(X_{i}+2*D_{i}-K_{i}\right)}{S_{i}}+1. \end{array}$$

In (1), *X*_*i*_ refers to the size of *i* in the input layer; *Y*_*i*_ accords to the size of *i* in the output layer; *K*_*i*_ expresses the size of the convolution kernel; *S*_*i*_ stands for the step length in the convolution process; *D*_*i*_ is the length of extension on the length of side.

#### 2.2.2. Expression of Time Sequence Features of GCMPs

The present work does not track the player's trajectory when identifying events in basketball video, but excavates the temporal characteristics between GCMPs based on LSTM and analyzes the continuous frame events [16, 17].

If the optical flow corresponding to the video frame of the video with a length of *T*+1 is GCMPs expressed by the calculation between adjacent video frames, then the spatial features of GCMPs are extracted by the CNN model. Finally, the spatial features of GCMPs are processed by the LSTM model, and the prediction results are output by temporal expression [18–20]. Equation (2) displays the calculation process.

(2) $$\begin{array}{c} \left\{\begin{array}{c} h_{1}=F_{w}\left(x_{1},h_{0}\right)=F_{w}\left(x_{1},0\right),\\ \begin{array}{c} h_{2}=F_{w}\left(x_{2},h_{1}\right),\\ \cdots \end{array}\\ h_{T}=F_{w}\left(x_{T},h_{T-1}\right), \end{array}\right. \end{array}$$

In (2), *x*_*T*_ denotes the input of the LSTM unit at time *T*, namely, the input of CNN; *w* refers to the weight matrix. *h*_*T*−1_ will be output, when weight matrix functions on the hidden layer at time *T* − 1; *x*_*T*_ will be input at time *T* when the hidden layer operates; *h*_*T*_ will be output to transmit to the hidden layer. Hence, videos should be processed in a timing order.

*N* represents the number of categories, and (3) expresses its responding value, when the neuron *n* responds to the neuron *t*.

(3) $$\begin{array}{c} s_{tn}=\sum {}_{i=1}^{256}h_{ti}*w_{in}+b_{n}. \end{array}$$

Equations (4) and (5) present the predicted results.

(4) $$\begin{array}{c} p_{tn}=\frac{\exp\left(s_{tn}\right)}{\sum {}_{n=1}^{N}\exp\left(s_{tn}\right)}, \end{array}$$

(5) $$\begin{array}{c} G=\frac{\sum {}_{t=1}^{T}\left(p_{t1},p_{t2},\ldots ,p_{tN}\right)}{T}. \end{array}$$

In (4) and (5), *G* refers to the final predicted results vector of the video, and *p*_*t*1_, *p*_*t*2_,…, *p*_*tN*_ represents the predicted results matrix with frame as *t*. The average score of *T* frames of videos needs to be obtained. And the event type of the video can be determined after judging the obtained results according to category.

### 2.3. Segmentation of Players in the Video by FCN-CNN

Figure 4 demonstrates the FCN-CNN algorithm to segment players in video, which is designed here.

#### 2.3.1. Clustering Segmentation of Superpixels

To ensure the local consistency of video pixel features and improve the learning efficiency of players, the mean shift method is used to segment the subsequent players based on superpixels when clustering the video pixels of the detected players, so that the complexity of the algorithm is effectively reduced.

Clustering based on feature space can realize the preprocessing of superpixels [21, 22]. When using the mean shift algorithm, the input value is a five-dimensional space containing two-dimensional physical coordinates (x, y) and three-dimensional color coordinates (l, *u*, v). In the process of algorithm operation, it is necessary to calculate the average value of pixels in the image for offset. Then, the pixels are moved according to the average value, and the moving points are used as the reference points of the image to repeat this process until the image reaches convergence.

After moving the pixels, labels will be assigned to each pixel. If the labels assigned to the two pixels are the same, it indicates that the visual characteristics of the two pixels have a certain similarity. Therefore, the color intensity, texture, and other characteristics are similar, contained in the superpixels. After the superpixels clustering segmentation of the image, the local consistency of the players can be guaranteed, and the wrong segmentation of the ambiguous pixels on the edge of the players can be effectively avoided [23–25].

#### 2.3.2. FCN Presegmentation

Here, FCN is used in the presegmentation of players, and Figure 5 bespeaks its structural framework.

Compared with the traditional CNN, the full CNN has a wider application range in the field of image segmentation. It can segment the semantic features in the image. Different from the neural network, the full CNN can classify all the pixels contained in the image when classifying the image, while the CNN classifies the image as a whole. Therefore, compared with the neural network, the extended full CNN has a better segmentation effect on the image [26–28].

To make the final image consistent with the size of the input image, it is necessary to conduct deconvolution according to the output image. If the size of the feature map is 1/32, it is upsampled, and its step length is 32. The image obtained by deconvolution is only the feature in the convolution layer 5. At this time, the information in the image is not complete and rough. Therefore, this method is not very suitable for image segmentation.

To solve the above problems existing in the images, it is necessary to supplement the details of the image. This process can be realized by fusing the image features obtained by convolution layer 4 and the results after upsampling of convolution layer 5. Then, the upsampling results are deconvoluted and fused with the image features obtained by convolution layer 3 and upsampled. Finally, the original image is obtained.

#### 2.3.3. CNN Optimized Segmentation

Since the full CNN may have a judgment error in the classification of super pixels regions, the results can be supplemented and predicted by the CNN. To improve efficiency, only the key pixels can be selected when the superpixels region features are expressed, and the calculation amount of the whole process can be greatly reduced by judging the selected key pixels through a convolution neural network [29, 30].

The process of optimizing segmentation with a CNN is as follows: at first, the superpixel to be processed is transformed into a one-dimensional vector. Since the texture, color, and visual features of the pixels contained in a superpixel have strong similarity, when superpixel features are represented, the odd number of *n* more important pixels can be selected to replace it [31].

When selecting the pixels, the random method or the consistent interval method can be used. When the key points are selected, the selected points may fall to the edge. Simultaneously, the pixel can not only express the player's behavior but also express the background. To avoid this problem, the superpixel is corroded before selecting the key points, as shown in

(6) $$\begin{array}{c} K\left(I\right)=\left\{b|L_{b}\subset I\right\}. \end{array}$$

In (6), *I* refers to the superpixel to be corroded; *L* represents the structural unit; *L*_*b*_ means translating the structural unit to the point *b*. If the superpixel to be corroded includes *L*_*b*_, point *b* will be marked, and the set it forms is named the results of *I* being corroded by *L*.

The *n* important pixels selected in the above process are taken as the center of the square subblock, and its edge length is changed to 57 after being clipped. The clipped subblock is taken as the input of the convolutional neural network to identify the characteristics of the important pixels. Finally, the characteristics of the selected important pixels are processed by voting. If (*n*+1)/2 important pixels are identified as a player after the judgment of the CNN, the whole region can be determined as a player, and vice versa.

## 3. Analysis of Types of Players' Postures

Figure 6 presents three main postures in the basketball game videos, which are standing, moving, and jumping.

Figure 6 demonstrates that, in the video analysis of basketball game, “jumping” refers to the action behavior of players when they take the ball to shoot, “moving” refers to the action behavior of players running sideways, and other action behaviors of players are called “standing.”

### 3.1. Experimental Settings

#### 3.1.1. Experimental Settings in the Basketball Video Events Analysis

To analyze the effectiveness of the classification of basketball game videos after integrating professional knowledge and global group movement patterns proposed here, the present work will conduct experimental analysis on National Collegiate Athletic Association (NCAA), China Basketball Association (CBA), and National Basketball Association (NBA) game videos.

In the experiment, the video segments of semantic events in the NCAA dataset are expanded according to a certain length, and then the NCAA + dataset is obtained. Hence, there is no difference between the video segments of semantic events in the two datasets [32, 33]. In the present work, 250 basketball games videos are selected as the samples of the experiment here. Among them, 50 basketball games videos are used as the test set 1 of this experiment, and their data are used as the training set. Then 9407 and 2279 video segments of semantic events are selected as training set and test set 1, respectively. There are 11 categories of semantic events, including steals, dunking success/failure, other two-point shooting success/failure, layup success/failure, penalty success/failure, and three-point shot success/failure. Besides, test set 2 is also set, which concludes two NBA and CBA games [34].

#### 3.1.2. Experimental Settings of Estimation on Individual Player's Postures

The validity of the FCN-CNN method is verified in the following. The estimation indexes are “time” and “difference in pixels” when segmenting the players' images in the video. Equation (7) illustrates the calculation of the accuracy of the pixels.

(7) $$\begin{array}{c} P_{\text{pixel}}={\left\|L-L{}^{\prime }\right\|}^{2}. \end{array}$$

In (7), *L* refers to the segmentation label to be tested; *L*′ represents the real data label.

The final result is obtained by comparing CNN method, SP-CNN method, FCN8s method, and FCN-CNN method.

## 4. Experimental Results and Analyses

### 4.1. Experimental Results and Analyses of Events in the Basketball Game Videos

The number of semantic events in test set 1 is shown in Figure 7.

Figure 8 presents the number of events of each type in test set 2.

The purpose of this experiment is to classify six types of important basketball events, including stealing, dunking, other two-point shots, shooting, free throw, and three-point shots. In this experiment, the time of the beginning of the events is defined as the time when basketball is separated from the player's hands, and the end time is defined as when basketball touches the basketball board.

#### 4.1.1. Validity of GCMPs

Important events are classified by whether there are GCMPs or not, and their classification accuracy is compared, to verify the effectiveness of GCMPs.  Figure 9 displays the experimental results.

Figure 9 implies that the classification accuracy of the free throw is significantly improved with GCMPs. Besides, there is a certain improvement in that of other important events such as a layup, 2-pointer, and dunk. The mean is 49.65% of the classification accuracy of the none-GCMPs events, and it is 68.11% of the GCMPs events, meaning that the average classification accuracy of events is improved by 18.46%. Hence, GCMPs are assumed to be helpful to improve classification accuracy.

#### 4.1.2. Validity of the Two-Stage Classification Method

It is found in the related works of literature that, besides layup and other 2-pointer, there is no significant relevance among other important events in the event-occ video sections.  Figure 10 bespeaks the classification results of the important events, which are according to GCMP_DF_SVF features extracted from the experimental videos.

Figure 10 reveals that when the event-occ video segments are classified based on GCMP_DF_SVF, the accuracy is not high, especially for the prediction results of dunking and layup, which are only 19.35% and 22.9%. After calculation, the average accuracy of the prediction results of each event turns out to be 58.22%.

A test is made on the two-stage classification algorithm proposed here. At first, the features of event-occ video segments are extracted based on GCMP_DF_SVF, and then the five types of event classification of video segments are realized, whose results are shown in Figure 11.

To classify the layup and other two-point ball events, the GCMP_DF_SVF feature of the preevent video segment is extracted based on GCMPs.  Figure 12 displays the results.

The preevent video segment is used for the analysis of other two-point shots and layups. At this stage, the accuracy of layup and other two-point ball events can reach 48.96% and 85.81%, respectively.

Figure 13 presents the emerging results of classification results of events in event-occ video sections and preevent video sections.

Compared with the event-occ video segment classification results based on GCMP_DF_SVF, it is found that, after emerging the two stages, the prediction accuracy has been significantly improved, especially for the two types of events on the basketball and other 2-pointers. The prediction accuracy sees an improvement of the basketball event by 21.26%, and the prediction accuracy of the other 2-pointers sees an increment by 6.41%. The conclusion is that the two-stage classification method based on event-occ proposed here can effectively improve the classification efficiency of events.

#### 4.1.3. Validity of Introducing the Professional Knowledge

To evaluate the validity of introducing the professional knowledge, three groups of comparative experiments are carried out on the data set NCAA+. The test set 1 is not introduced with professional knowledge, test set 2 is introduced with partial professional knowledge, and test set 3 is introduced with full professional knowledge.  Figure 14 displays the experimental results.

Figure 14 indicates that, except for the other 2-pointers failure events, the prediction accuracies of Experiment 3 and Experiment 2 for the remaining events are significantly higher than that of Experiment 1. Simultaneously, Figure 14(b) suggests that, compared with Experiment 1, there is an increment of 9.32% in the average prediction accuracy of Experiment 2 with partial professional knowledge. Furthermore, there is an increment by 10.74% in the average prediction accuracy of Experiment 3 with full professional knowledge compared with Experiment 2. The conclusion is that the integration of professional knowledge is conducive to the improvement of algorithm performance.

### 4.2. Experimental Results of Prediction on Players' Postures

#### 4.2.1. Distribution and Changes of Players' Posture in Different Events

To analyze the changes of players' postures at different time, present work analyses the posture of players in two complete basketball games. The video segments of six types of events are analyzed, including snatching, dunk, layup, the other two points, penalty, and three-point. Analysis is made on the video segments of the above events.  Figure 15 denotes the analysis results of the players' postures.

Figure 15(a) indicates that players' postures are standing and moving in the “snatching,” and no player jumps in this event.  Figure 15(b) suggests that players' postures are jumping and shooting in the “dunking,” and the other player keeps standing or moving in this event. Besides, the duration of the event is 14 seconds.  Figure 15(c) implies that there many players postures are standing, and few players are jumping or moving.  Figure 15(d) indicates that there are many players in an active status in the layup, and few players are standing.  Figure 15(e) illustrates that, at the beginning of the three-pointer, each of the pitcher and the defender has a jump attitude, and when the ball is put, the status of the jumper turns 0. Hence, in different basketball events, the players' postures are also quite different.

#### 4.2.2. Segmentation Results of Players

Figure 16 demonstrates the analytical results of the performance of CNN, SP-CNN, FCN8, and FCC-CNN4 segmentation methods.

The player segmentation test phase is carried out on Nvidia Tesla K40 C GPU. CNN predicts that the time of a key pixel feature is 0.04 seconds. It is counted that the average number of pixels of 100 players is 17666, so the time consumption of CNN method is 706.64 seconds. In the test stage of Superpixel-Convolutional Neural Network (SP-CNN), if five key points are selected at equal intervals for each superpixel, it takes 0.2 seconds to process a superpixel. However, in the test stage, it takes 20 seconds to set the number of superpixels of players to 100; that is, it takes 20 seconds to segment through SP-CNN. The average time for FCN8s to realize player segmentation is 1.02 seconds. Compared with CNN in the field of segmentation, FCN has great advantages in speed, but it lacks accuracy. In the testing stage by FCN-CNN method, it is found that the average number of remaining superpixels after FCN8s preprocessing is 20; that is, the CNN optimization processing takes 4 seconds at this stage and the FCN-CNN segmentation method takes 5.02 seconds.

Figure 16 reveals that the gap between FCN-CNN, SP-CNN, and CNN is not particularly obvious only in terms of segmentation accuracy, but in terms of segmentation time, FCN-CNN method based on superpixel guidance has great advantages.

#### 4.2.3. Prediction Results of Players' Postures

Data of 639 basketball players are recognized as the test set and data of other 2590 basketball players is recognized as a training set in this experiment.  Figure 17 illustrates the number of players of according postures in the training set and testing set.

In the experiment, the batch size is set as 128; that is, the data of 128 players will be processed for each successive iteration. The initial learning rate is set to 0.001, and the learning rate will decline by half after 100 iterations. When the number of iterations reaches 15000, the accuracy of the model will reach a fixed value. Based on the optimal model, data of 639 players in the test set are tested, whose results are displayed in Figure 18.

Figure 18 indicates that the method can make a rather highly accurate classification on moving postures of players, with an accuracy of 83.33%, while it makes the lowest accurate classification on standing postures, with an accuracy of 75.31%. In the prediction on mobile postures of 192 players, 160 players' postures are correctly predicted. In the remaining 32 players, 24 players' postures are mispredicted as jumping, and postures of the rest of them are mispredicted as standing. In the prediction of postures of 204 players, postures of 169 players are correctly predicted, and in the rest of the postures of 35 players, 5 of them are mispredicted as moving and the other is mispredicted as standing. In the prediction of postures of 243 standing players, 183 of them are correctly predicted. In the rest 60 players, 35 of them are mispredicted as moving, and the rest are mispredicted as jumping.

## 5. Conclusions

It has been a hot topic of scientifically managing the videos related to sport game events, along with the widespread of these videos on the internet. In the past, to analyze basketball game videos, broadcasters need to distinguish different events of players based on audio features and text. It is a big waste of manpower and material resources, and the traditional method has a high error rate due to some subjective factors.

The present work studies the event classification of basketball games in multiplayer videos. At first, the group and global motion characteristics are extracted to express the accorded event. A complete basketball game video is divided into three parts: preparation, occurrence, and end. The present work proposed a basketball event classification method based on global group motion mode and domain knowledge fusion. Subsequently, a target segmentation method based on FCN-CNN is proposed to realize the automatic segmentation of player area through the detection of players through SSD network. The segmentation algorithm includes superpixel clustering, presegmentation of players based on FCN8s, and finally segmentation optimization of players through CNN according to the constraints of superpixel. Based on the segmented player area, the current work continues to estimate the individual posture of the player, from the statistics of the distribution of the player's posture in different events to the estimation of the player's posture based on the deep learning CNN. Finally, the misjudgment of the player's posture is analyzed in detail.

The current work analyzes the basketball game video in multiperson cooperative sports video, studies the semantic event classification of basketball game video, and aims to propose an event analysis method of basketball sports video based on deep learning and promote the rapid development of basketball and even sports. Although the experimental results of the proposed method are higher than other classification results in the field of basketball video event classification, there is still a certain gap in the future practical application. In the future work, the exploration will be carried out from the following aspects: for the expression of players' movement patterns, the optical flow graph calculation model based on deep learning can be used to extract the players' group movement patterns from the complex movement patterns of sports video pictures. This can effectively suppress the interference of irrelevant information in the scene, such as audience area, field picture and lens motion, to improve the learning efficiency of the model for the key information in the scene.

## Figures and Tables

**Figure 1:** Total framework of multidomain knowledge and GCMPs.

**Figure 2:** Framework diagram based on GCMPs event classification.

**Figure 3:** CNN framework to learn spatial features of GCMPs.

**Figure 4:** Players segmentation framework based on FCN-CNN.

**Figure 5:** The structural framework of prsegmentation of players.

**Figure 6:** Demonstration of player's posture. (a) Jumping; (b) standing; (c) moving.

**Figure 7:** Classification and number of events in the test set 1.

**Figure 8:** Classification and number of events in the test set 2. (a) NBA games; (b) CBA games.

**Figure 9:** Analytical results of the validity of GCMPs.

**Figure 10:** Classification results based on GCMP_DF_SVF. (a) Prediction results; (b) accuracy.

**Figure 11:** Classification results of five types of the event of event-occ video segments.

**Figure 12:** Classification results of events in preevent video sections.

**Figure 13:** Classification results of emerging the two stages.

**Figure 14:** Influence of professional knowledge on the performance of algorithms. (a) Comparison of 3 groups of the accuracy; (b) comparison of the average accuracy.

**Figure 15:** Statistical results of players' postures: (a) snatching; (b) dunking; (c) other two-pointers; (d) layup; (e) penalty; (f) three-pointer.

**Figure 16:** Comparison between the performance of segmentation methods. (a) Comparison of accuracy; (b) comparison in duration.

**Figure 17:** Distribution of data of players. (a) Training set; (b) test set.

**Figure 18:** Test results. (a) Test results of players' postures; (b): accuracy of prediction.

## Data Availability

The research data used to support the findings of this study are included within the article.
